# Suppression of growth, migration and invasion of highly-metastatic human breast cancer cells by berbamine and its molecular mechanisms of action

**DOI:** 10.1186/1476-4598-8-81

**Published:** 2009-10-01

**Authors:** Shan Wang, Qian Liu, Ying Zhang, Ke Liu, Pengfei Yu, Kun Liu, Jinling Luan, Huiying Duan, Zhaoqiao Lu, Fengfei Wang, Erxi Wu, Kazumi Yagasaki, Guoying Zhang

**Affiliations:** 1 Laboratory of Molecular Pharmacology, School of Pharmacy, Yantai University, No 30, Qing Quan Lu, Lai Shan Qu, Yantai, Shandong Province 264005, China; 2 Clinical Medicine, Clinical College of Anhui Medical University, No 15, Feicuilu, Hefei, Anhui Province 230601, China; 3 Department of Pharmaceutical Sciences, North Dakota State University, Fargo, ND, 58105, USA; 4 Department of Applied Biological Science, Tokyo Noko University, Saiwai-cho 3-5-8, Fuchu, Tokyo 183-8509, Japan

## Abstract

**Background:**

Breast cancer is the second leading cause of cancer related deaths among females worldwide. Berbamine (BER), a kind of bis-benzylisoquinoline alkaloid, has been used to treat clinical patients with inflammation and cancer for many years in China. The purpose of this study is to investigate the activity of BER against highly-metastatic human breast cancer and its molecular mechanisms of action.

**Results:**

In our study, we found that BER inhibits growth of highly-metastatic human breast cancer cell lines MDA-MB-231 and MDA-MB-435S cells dose-dependently and time-dependently. The sera from BER-treated rats suppress the growth of MDA-MB-231 cells. BER shows synergistic effects with some existing anticancer agents such as trichostatin A (TSA, the histone deacetylase inhibitor), celecoxib (the inhibitor of COX-2), and carmofur against the growth of MDA-MB-231 cells. BER also displays the strong activity of inducing apoptosis in both estrogen receptor-negative MDA-MB-231 cells and estrogen receptor-alpha-positive MCF-7 breast cancer cells, but not in normal human mammary epithelial cell line MCF10A. BER down-regulates anti-apoptotic protein Bcl-2 levels and up-regulates pro-apoptotic protein Bax expressions in MDA-MB-231 and MDA-MB-435S cells. BER also has synergistic effects with anticancer agents trichostatin A, celecoxib and/or carmofur on reducing Bcl-2/Bax ratios and VEGF secretions in MDA-MB-231 cells. In addition, BER significantly suppresses cell migration and invasion, as well as decreases pro-MMP-9/pro-MMP-2 activation in breast cancer cells. Furthermore, BER suppresses Akt and nuclear factor *κ*B signaling by reducing the phosphorylation of c-Met and Akt, and inhibiting their downstream targets such as nuclear factor *κ*B p-65, Bcl-2/Bax, osteopontin, VEGF, MMP-9 and MMP-2 on protein and/or mRNA levels in breast cancer cells.

**Conclusion:**

Our findings have showed that BER suppresses the growth, migration and invasion in highly-metastatic human breast cancer cells by possibly inhibiting Akt and NF-*κ*B signaling with their upstream target c-Met and downstream targets Bcl-2/Bax, osteopontin, VEGF, MMP-9 and MMP-2. BER has synergistic effects with anticancer agents trichostatin A, celecoxib and carmofur on inhibiting the growth of MDA-MB-231 cells and reducing the ratio of Bcl-2/Bax and/or VEGF expressions in the cancer cells. These findings suggest that BER may have the wide therapeutic and/or adjuvant therapeutic application in the treatment of human breast cancer and other cancers.

## Background

Breast cancer is the second leading cause of cancer-related deaths among females in the United States [1]. Its rate in China and other Asian countries is also increasing rapidly [2,3]. To find novel natural compounds with low toxicity and high selectivity for killing cancer cells is an important area in cancer research. To date, chemotherapy has been the most frequently used treatment for breast cancer and other cancers. However, some normal cells are destroyed as well by this method of treatment. Due to their wide range of biological activities and low toxicity in animal models, some natural products have been used as alternative treatments for cancers including breast cancer. Berbamine (BER) is a naturally occurring small-molecule compound from Traditional Chinese Medicine (TCM) *Berberis amurensis *(xiaoboan). In China, BER has been used to treat the clinical patients with inflammation and various cancers including breast cancer, hepatoma, leukemia for many years. BER is also a clinical drug to treat the patients with low levels of white blood cells, which are caused by chemotherapy and/or radiotherapy. The chemical structure of BER is shown in Fig. 1A. BER-induced apoptosis and growth inhibition of human leukemia HL-60 and K562 cell lines without cytotoxicity to normal hematopoietic cells [4-6]. It induced caspase-3-dependent apoptosis of leukemia NB4 cells via survivin-mediated pathway [7]. BER also caused apoptosis and cell cycle arrest, and led to loss of mitochondrial membrane potential and activated caspase-3 and caspase-9 in human hepatoma cells [8]. However, whether or not BER has inhibitory activities against highly-metastatic human breast cancer cells is unclear. In this study, we investigated the effects of BER on growth, migration and invasion of highly-metastatic human breast cancer cells and its molecular mechanisms of action. We showed that BER inhibited the growth, migration and invasion of the highly-metastatic human breast cancer cells as well as induced the apoptosis in the cancer cells. Such anti-cancer activities of BER involved suppression of Akt and NF-*κ*B signaling and its upstream and downstream targets by reducing expressions of the related proteins and mRNA as well as pro-MMP-9/pro-MMP-2 activation in the cells.

**Figure 1:** ***In vitro*/*ex vivo *growth inhibition of highly-metastatic human breast cancer cell lines by berbamine (BER)**. (A) The chemical structure of berbamine. Growth inhibition of highly-metastatic human breast cancer cell lines MDA-MB-231 (B) and MDA-MB-435S (C) cells after treatment for 24 hour (h), 48 h and 72 h with 1-80 μM BER (B, left panel) or the sera (B, right panel) taken from rats (n = 6 for each group at different time points) at 0 h (as the control group), 1 h, 2 h and 3 h after oral administration of BER in rats, respectively. The cell growth was determined by MTT assay. (D) *In vitro *effects of BER and its synergistic anticancer agents on growth of MDA-MB-231 cells. The cells were treated for 48 h with the indicated concentrations of BER (B, 1- 40 μM), celecoxib (S, 10-80 μM), trichostatin A (T, 12.5-100 μg/L), carmofur (KA, 40 mg/L), navelbine (NA, 5 nM), rosiglitazone (Ro1, 1 μM), lovastatin (Lo1, 1 μM), Ly294002 (LY, 12.5 and 25 μM), and Bay (5 μM) in the absence or presence of the synergistic anticancer agents S (20 and 40 μM), T (25 and 50 μg/L), KA (40 mg/L), LY (12.5 and 25 μM). The data are presented as the mean ± SD (Bar) for each group (n = 6). The figures (B, C and D) are the representative of 3 similar experiments performed. Comparison was made by two-way ANOVA followed by Bonferroni post hoc test to establish whether significant differences existed between the groups. *: *P *< 0.05, ***, *P *< 0.001. All statistical tests were two-sided. Values with different letters (a-i) differ significantly (*P *< 0.05). i/s, f/s and h/s represent the significant synergistic effects (*P *< 0.05) compared with the treatment with its individual compound alone. (i/s, *P *< 0.0001, two-way ANOVA; f/s, *P *< 0.001, two-way ANOVA; h/s, *P *< 0.001, two-way ANOVA).

## Results

### In vitro and ex vivo inhibition of growth in human breast cancer cells by BER and its synergistic effects with anticancer agents in dose- and time-dependent manners

We first investigated the effects of BER on the growth of highly-metastatic human breast cancer cell lines, MDA-MB-231 and MDA-MB-435S. The growth of both human breast cancer cell lines was inhibited by BER after the cells were treated with BER at the concentrations of 1 to 80 μM for 24, 48 and 72 h, respectively. The IC_50 _values at 24, 48 and 72 h were 51.6, 32.5, and 13.7 μM for MDA-MB-231 cells and (42.3 μM, 34.3 μM, and 25.0 μM) for MDA-MB-435S cells, respectively (Fig. 1B and 1C). Furthermore, the sera collected at 1 h and 2 h from BER-treated rats significantly suppressed the growth of MDA-MB-231 cells after the cells were treated with the sera for 48 and 72 h, respectively, as compared with 0 h sera taken at 0 h from rats. The 3 h sera from BER-treated rats did not show significant inhibition of the cancer cell growth. The peak time of the *ex vivo *inhibition of the cell growth by the rat sera was between 1 h and 2 h after the rats were administered orally with BER (Fig. 1B). In addition, BER showed the synergistic effects with the existing anticancer agents celecoxib (the inhibitor of COX-2), trichostatin A (TSA, the histone deacetylase inhibitor), and carmofur (KA or K) against the growth of MDA-MB-231 cells, which enhanced inhibitory rate of the cancer cell growth more than twice. As the positive control, the anticancer agents celecoxib, trichostatin A, carmofur, rosiglitazone, lovastatin, navelbine, Ly294002 (the inhibitor of PI3K/Akt) and Bay (the inhibitor of NF-*κ*B) showed significant inhibition of the growth of MDA-MB-231 cells (Fig. 1D).

### The strong induction of apoptosis in both estrogen-receptor negative/highly-metastatic human breast cancer cells and estrogen receptor-alpha-positive human breast cancer cells, rather than in normal human mammary epithelial cells by BER

Next, we investigated effects of BER on the apoptosis of both human breast cancer cell lines and normal human mammary epithelial cell line. Flow cytometric analysis further confirmed that BER at concentrations of 20 μM, 40 μM, and 60 μM displayed dose-dependent induction of apoptosis in both estrogen-receptor negative and highly-metastatic human breast cancer cell line MDA-MB-231 cells, and the estrogen receptor-alpha-positive MCF-7 cells after the cells were treated for 48 h with BER. Whereas, such treatment with the same concentrations of BER (except 60 μM) did not show strong toxicity to the human mammary epithelial cell line MCF10A (Fig. 2A and 2B).

**Figure 2:** **The strong induction of apoptosis in both estrogen-receptor negative and estrogen receptor-alpha-positive breast cancer cells**. FACS analysis (A) of the cell cycles and apoptosis in estrogen-receptor negative cell line MDA-MB-231 and estrogen receptor-alpha-positive breast cancer cell line MCF-7 as well as normal human mammary epithelial cell line MCF-10A after the cells were treated for 48 h with BER at the indicated concentrations. The percent apoptosis(cells in subG_1 _phase) in the cells treated by BER are summarized in (B).

### Up-regulation of Bax protein levels and down-regulation of Bcl-2 protein expressions in highly-metastatic human breast cancer cells by BER and its synergistic effects with anticancer agents

Further study on the mechanisms of action of BER induced apoptosis in the highly-metastatic human breast cancer cells showed that the expressions of anti-apoptotic protein Bcl-2 were down-regulated and the levels of pro-apoptotic protein Bax were up-regulated in both MDA-MB-231 and MDA-MB-435S cells after the cells were treated for 48 hours with BER at concentrations of 40 μM and 60 μM (Fig. 3A and 3B). In addition, BER displayed the synergistic effects with anticancer agents celecoxib and trichostatin A on reducing Bcl-2 protein expression and increasing Bax protein level, which twice reduced the ratio of Bcl-2 and Bax levels in MDA-MB-231 cells (Fig. 3C).

**Figure 3:** **Effects of BER with its synergistic anticancer agents on Bcl-2/Bax protein expressions in MDA-MB-231 cells**. Western blot analysis of Bcl-2 (A) and Bax (B) expressions in whole-cell lysates of MDA-MB-231 (left panel) and MDA-MB-435S (right panel) cells treated for 48 h with BER at the indicated concentrations; (C) Reduction of Bcl-2/Bax ratio in MDA-MB-231 cells by BER and its synergistic anticancer agents celecoxib and trichostatin A. The cells were treated for 48 h with the indicated concentrations of BER (B, 20 μM), celecoxib (S, 20 μM), trichostatin A (T, 50 μg/L), Ly 294002 (LY, 25 μM), and Bay (5 μM) in the absence or presence of its synergistic anticancer agents S (20 μM) and T (50 μg/L). The expressions of Bcl-2 and Bax in MDA-MB-231 were analyzed by Western blotting. In the (A) and (B), the density of the band (normalized to β-actin) shown as mean ± SD (Bar) is relative to that of 0 as the control (designated as 100%). In the (C), the ratio of Bcl-2 and Bax, (the ratio of relative density of each band normalized to β-actin), shown as mean ± SD (Bar) is relative to that of 0 (0.1% DMSO vehicle) as the control (designated as 1.0). For one experiment, 3 assays were carried out and only one set of gels is shown. Comparison was made by two-way ANOVA followed by Bonferroni post hoc test to establish whether significant differences existed between the groups. *: *P *< 0.05, **, *P *< 0.01. Values with different letters (a-e) differ significantly (*P *< 0.05). e/s+ represents the significant synergistic effects (*P *< 0.05) compared with the treatment with its individual compound alone. Statistically significant synergistic effect on the Bcl-2/Bax ratio was observed in MDA-MB-231 cells treated with B20+S20 or B20+T50 compared with the individual B20, S20 or T50 treatment alone (B20+S20, *P *< 0.001, two-way ANOVA; B20+T50, *P *< 0.001, two-way ANOVA).

### Suppression of migration and invasion as well as reduction of pro-matrix MMP-9/MMP-2 activation in highly-metastatic human breast cancer cells by BER

Cancer cell migration and invasion play very important roles in cancer metastasis. So, we further studied the effects of BER on migration and invasion as well as the related pro-MMP-9/pro-MMP-2 activation in MDA-MB-231 cells. Migration assay by fibronectin-coated transwell chamber showed that BER at low concentrations of 10 μM and 20 μM significantly suppressed the migration of MDA-MB-231 cells with the inhibition rate of 43.8% and 59.2%, respectively after the cells were treated for 6 h with BER (Fig. 4A). Invasion assay in Matrigel-coated transwell chamber indicated that BER at low concentrations of 10 μM and 20 μM significantly suppressed the invasion of MDA-MB-231 cells with the inhibition rate of 40.0% and 54.5%, respectively after the cells were treated for 16 h with BER (Fig. 4B). The gelatin zymography analysis further demonstrated that the activation of pro-matrix MMP-9 and pro-matrix MMP-2 in the supernatants of invading MDA-MB-231 cells was suppressed markedly by BER at 1 μM, 10 μM and 20 μM (Fig. 4C).

**Figure 4:** **Suppression of migration and invasion and pro-matrix MMP-9/MMP-2 activation in MDA-MB-231 cells by BER**. MDA-MB-231 cell migration (A) was examined in the presence of BER at the indicated concentrations for 6 h in upper chamber of the fibronectin-coated transwell chamber (serum-free). The right panels show the propidium iodide-stained MDA-MB-231 cells migrating through fibronectin-coated transwell chamber. The cells were treated 6 h with the 0 (A1: vehicle as the control) and 20 μM BER (A2). In the (B), MDA-MB-231 cell invasion was examined in the presence of BER at the indicated concentrations for 16 h in upper chamber of the Matrigel-coated transwell chamber (serum-free). The right panels show the propidium iodide-stained MDA-MB-231 cells invading through Matrigel-coated transwell chamber. The cells were treated 16 h with the 0 (B1: vehicle as the control) and 20 μM BER (B2). Relative migration (%) ± SD (Bar) and relative invasion (%) ± SD are shown for the indicated BER concentrations and the 0 (vehicle) is the control. (C) Inhibition of pro-matrix MMP-9/MMP-2 activation in supernatants of invading MDA-MB-231 cells by BER. MDA-MB-231 cells were cultured for 16 h in upper chamber of the Matrigel-coated transwell chamber (serum-free) in the presence of BER at 0, 1 μM, 10 μM, and 20 μM, respectively. The activation (*M*r 72,000 and *M*r 92,000 gelatinase activities) of MMP-9/MMP-2 zymogens (z-MMP-9/z-MMP-2) in the supernatants of invading MDA-MB-231 cells mentioned in (B) was determined by gelatin zymography analysis. Values (the relative activation of MMP-9/MMP-2 zymogens) are shown as mean ± SD of 3 runs (n = 3) for each sample, only one set of gels is shown. The figures (A, B and C) are the representative of 3 similar experiments performed. Statistical analysis was done using the ANOVA and Bonferroni test. *: *P *< 0.05, **, *P *< 0.01 (n = 6).

### Suppression of phosphorylation of Akt and c-Met, expressions of NF-*κ*B and secretions of osteopontin and VEGF proteins as well as mRNA levels of MMP-2 and MMP-9 in highly-metastatic human breast cancer cells by BER

Phosphoinositide 3-kinase (PI3K)/Akt and NF-*κ*B signaling pathways are associated with the growth, migration, invasion, angiogenesis and metastasis in cancer progression [9-18]. PI3K plays a central role in a diverse range of cellular responses including cell growth and survival [19,20]. Akt (also named protein kinase B) is a downstream signal of PI3K and a 60 KD serine/threonine kinase and is also a critical mediator of survival signals to protect cells from apoptosis [21,22]. Activation of the PI3K/Akt pathway in response to cytokines leads to phosphorylation and activation of the nuclear factor NF-*κ*B p65/RelA subunit, which regulates expression of anti-apoptotic genes [23,24]. Activation of NF-*κ*B blocks the apoptotic response in a variety of cells, including breast cancer [25]. To further clarify the mechanisms of action of BER suppressing the growth and reducing the cell migration and invasion in MDA-MB-231 cells, we investigated the effects of BER on p-Akt, NF-*κ*B, and their upstream target c-Met and downstream targets OPN, VEGF, MMP-9 and MMP-2 in MDA-MB-231 cells. Western blot analysis confirmed that BER at the concentrations of 1-60 μM significantly suppressed the phosphorylation (Ser473) of Akt (Fig. 5A) and NF-*κ*B p-65 expressions (Fig. 5B) in MDA-MB-231 cells. In addition, BER at the concentrations of 5-60 μM displayed significant reduction of the phosphorylation of c-Met in MDA-MB-231 cells (Fig. 5C). Furthermore, ELISA analysis indicated that BER at concentrations of 40 μM and 60 μM markedly reduced the secretions of osteopontin (OPN), a metastasis-associated protein in both MDA-MB-231 and MDA-MB-435S (Fig. 6A) cells after the cells were treated for 16 h with BER. There have been studies showing that MDA-MB-231 cells can secrete VEGF [26,27]. The present study indicated that BER at concentrations of 10-40 μM dose-dependently decreased the VEGF secretion in MDA-MB-231 cells. More importantly, BER displayed the synergistic effects with anticancer agents trichostatin A and carmofur on reducing the secretions of VEGF in MDA-MB-231 cells. Furthermore, the anticancer agents celecoxib, rosiglitazone, lovastatin, Ly294002 and Bay showed the reduction of the VEGF secretions in the breast cancer cells (Fig. 6B). RT-PCR detection demonstrated that BER at 40 μM and 60 μM dramatically reduced the mRNA levels of MMP-2 (Fig. 7A) and MMP-9 (Fig. 7B) in MDA-MB-231 cells after the cells were treated for 16 h with BER.

**Figure 5:** **Suppression of phosphorylation of Akt and c-Met as well as NF-*κ*B expression in MDA-MB-231 cells by BER**. The cells were treated with BER at the indicated concentration and the 0 (vehicle) is the control. Equal amounts of protein from total cell lysates were separated by SDS-PAGE, and Western blot analysis of p-Akt (A), p-c-Met (C) and NF-*κ*B (B) were done. For the analysis of phosphorylation of Akt and c-Met, the density of the band (normalized to Akt and c-Met, respectively) shown as mean ± SD is relative to that of 0 (vehicle) as the control (designated as 100%). For analysis of the NF-*κ*B p65 expression, the density of the band (normalized to β-actin) shown as mean ± SD is relative to that of 0 (vehicle) as the control (designated as 100%). Bay and LY (LY294.002) are the inhibitors of NF-*κ*B and PI3K/Akt, respectively. For one experiment, 3 assays were carried out and only one set of gels is shown. The phosphorylation of Akt and c-Met as well as NF-*κ*B p65 expression in MDA-MB-231 cells were significantly suppressed by BER. Statistical analysis was carried out using the ANOVA and Bonferroni test. *: *P *< 0.05 (n = 3). Values with different letters (a-c) differ significantly (*P *< 0.05).

**Figure 6:** **Reduction of secretions of osteopontin (OPN) and VEGF in MDA-MB-231 cells by BER**. (A) Reduction of OPN secretions in MDA-MB-231 (left) and MDA-MB-435S (right) cells by BER treatment. The cells were treated for 16 h with BER at the indicated concentration. The secreted OPN in the cell supernatants was analyzed by ELISA described in "Materials and Methods" section. (B) Reduction of VEGF secretions in MDA-MB-231 cells by BER and its synergistic anticancer agents carmofur (K) and trichostatin A (T). The 0 (0.1% DMSO vehicle) is the control. The cells were treated for 48 h with the indicated concentrations of BER (B, 10 μM, 20 μM, and 40 μM), celecoxib (S, 10 μM, 20 μM, 40 μM and 80 μM), trichostatin A (T, 25 μg/L and 50 μg/L), carmofur (K, 40 mg/L), rosiglitazone (Ro1, 1 μM), lovastatin (Lo1, 1 μM), Ly294002 (LY, 25 μM), and Bay (5 μM) in the absence or presence of its synergistic anticancer agents K (40 mg/L) and T (25 μg/L and 50 μg/L). The secreted VEGF in the supernatants of MDA-MB-231 cells was analyzed by ELISA described in "Materials and Methods" section. Values are shown as mean ± SD (bar) for the indicated concentration (n = 3). Comparison was made by two-way ANOVA followed by Bonferroni post hoc test to establish whether significant differences existed between the groups. *: *P *< 0.05, **, *P *< 0.01. Values with different letters (a-f) differ significantly (*P *< 0.05). e/s represents the significant synergistic effects (*P *< 0.001) compared with the treatment with its individual compound alone. Statistically significant synergistic effects on the VEGF secretions were observed in MDA-MB-231 cells treated with B20+K40+T25, B10+K40+T50, B20+K40+T50 compared with the individual B10, B20, T25, T50, and/or K40 treatment alone (e/s, *P *< 0.001, two-way ANOVA).

**Figure 7:** **Effects of BER on mRNA expressions of MMP-2 and MMP-9 in MDA-MB-231 cells**. The mRNA expressions were determined by semi-quantitative RT-PCR after the cells were treated for 16 h with BER at 0 (control), 40 μM and 60 μM. mRNA expression level was normalized to β-actin. For one experiment, 3 assays were carried out and only one set of gels is shown. The density of the band (normalized to β-actin) shown as mean ± SD is relative to that of the control (designated as 1.00). Statistical analysis was done using the ANOVA and Bonferroni test. Significant decreases in the mRNA expressions were observed in MMP-2 (n = 3) and MMP-9 (n = 3). **, *P *< 0.01, significant difference.

## Discussion

Abnormal growth and metastasis of cancer cells are regarded as the important biological characteristics of cancers. The presence of metastasis is the main cause of morbidity and mortality in millions of patients with cancer. During the complicated process of metastasis, the invasion of cancer cells is the most important and characteristic step. Clearly, an agent that could efficiently inhibit the growth, migration and invasion of cancer cells would be a hopeful candidate to suppress cancer progression and metastasis and thus it could reduce mortality. In the present study, we have demonstrated that BER suppressed the growth of highly-metastatic human breast cancer cell lines, MDA-MB-231 and MDA-MB-435S cells in dose- and time-dependent manners (Fig. 1B &1C). In addition, the sera taken at 1 h and 2 h from BER-treated rats displayed significant inhibitory effects against the growth of MDA-MB-231 cells *ex vivo *although 3 h sera did not show the significant inhibition (Fig. 1B). Whereas, we did not observe a significant effect on the cell growth when the cells were treated with the sera taken at 0 h, 1 h, 2 h, and 3 h from rats treated with water containing 0.9% NaCl (data not shown). There have been reports showing that the blood concentration of BER can be detected in rats and BER appeared in blood of rats 5 minutes after intravenous injection of BER [28]; BER appeared in blood and lung tissue of mice about 0.1-0.25 h after oral administration of BER [29]. These results suggest that BER has a certain bioavailability by oral administration and the BER and BER-induced changes of some factors in the sera may produce the effects on MDA-MB-231 cells growth. More importantly, BER showed the synergistic effects with anticancer agents celecoxib, trichostatin A, and carmofur against the growth of MDA-MB-231 cells, which enhanced the inhibitory rate of the cancer cell growth more than twice (Fig. 1D). These results further suggest that BER may have therapeutic and/or adjuvant therapeutic effects against the growth of human metastatic breast cancer cells. To understand the mechanisms of action of BER against the growth of the metastatic human breast cancer cells, we investigated the effects of BER on induction of apoptosis in the cancer and normal human mammary epithelial cells. The results indicated that BER strongly induced the apoptosis in both estrogen-receptor negative MDA-MB-231 cells, and estrogen receptor-alpha-positive MCF-7 breast cancer cells, but not in normal human mammary epithelial cell line MCF-10A (Fig. 2A and 2B). BER reduced the Bcl-2 protein expressions (Fig. 3A) and enhanced the Bax protein expressions (Fig. 3B) in the human breast cancer cells. Furthermore, BER displayed the synergistic effects with anticancer agents celecoxib and trichostatin A on reducing Bcl-2 protein expressions and increasing Bax protein levels, which twice reduced the ratio of Bcl-2 and Bax levels in MDA-MB-231 cells (Fig. 3C). These data suggest that induction of apoptosis of MDA-MB-231 cells is possibly one of important mechanisms of action of BER with celecoxib and trichostatin A against the growth of the human breast cancer cells.

Bcl-2 and its dominant inhibitor Bax are key regulators of cell growth and apoptosis. Overexpression of Bcl-2 enhances cell survival by suppressing apoptosis, but overexpression of Bax accelerates cell death. NF-*κ*B is a nuclear transcription regulator with a specific motif for Bcl-2 transcription [30-32]. The PI3K/Akt pathway acts as a survival (anti-apoptotic) signal and plays a key role in the regulation of apoptotic change in breast cancer cells. Akt can exert its anti-apoptotic effects in several different ways, such as negatively regulating pro-apoptotic factors, stimulating the NF-*κ*B survival pathway [23,24,33,34]. Activation of p-Akt and the NF-*κ*B/Bcl-2 pathway leads to inhibition of chemotherapy-induced apoptosis, which results in treatment resistance [25]. The Bax, Bcl-2, p-Akt and NF-*κ*B have become the important targets of action by anticancer agents [25,32,35-38]. Here, we have demonstrated that BER targets these factors in the human breast cancer cells. We have confirmed that BER inhibits the p-Akt and the NF-*κ*B/Bcl-2 pathway by suppressing the phosphorylation of Akt and NF-*κ*B expression in MDA-MB-231 cells (Fig. 5). This inhibition may contribute to the down-regulation of the levels of Bcl-2 protein and up-regulation of the levels of Bax protein in the human breast cancer cells. Such effects may be the important mechanisms of action of BER induced apoptosis and suppressed the growth of the breast cancer cells.

Increased OPN and VEGF levels, activation of p-c-Met and p-Akt, and enhanced expressions of NF-*κ*B and MMP-9/MMP-2 are associated with cancer cell growth, invasion, and metastasis as well as angiogenesis [9-18]. The receptor tyrosine kinase, c-Met and its ligand hepatocyte growth factor/scatter factor (HGF/SF), have become leading candidates for targeted cancer therapies. Inappropriate c-Met signaling through autocrine, paracrine, amplification, and mutational activation occurs in virtually all types of solid tumors, contributing to one or a combination of proliferative, invasive, survival, or angiogenic cancer phenotypes. c-Met and HGF/SF participate in all stages of malignant progression and represent promising drug targets in a variety of cancer types, including breast cancer [39]. The metastasis-associated protein, OPN, was reported to stimulate the motility and invasion of MDA-MB-231 cells through PI3K/Akt and NF-*κ*B signaling pathways [14]. VEGF is a key regulator of angiogenesis and VEGF expression correlates with tumor progression [40]. OPN and VEGF transcriptions were inhibited by abrogating NF-*κ*B activation [13,16]. OPN regulated pro-MMP-9 activation in cancer cells [15]. MMP-9 is a NF-*κ*B-regulated gene and is associated with invasion and metastasis, which is considered to be a therapeutic target of high priority [9,10]. MMP-2 was reported to play a direct role in OPN-induced cancer cell migration and invasion; OPN-stimulated MMP-2 activation occurred through NF-*κ*B mediation [12]. Therefore, the suppression of phosphorylation of c-Met and the blockage of PI3K/Akt and NF-*κ*B signaling pathways by the anticancer compounds could possibly inhibit the related downstream targets such as OPN, VEGF, MMP-9 and MMP-2, and thus suppress the cancer progression. Our present results have demonstrated that BER suppresses the phosphorylation of c-Met and Akt as well as NF-*κ*B p65 expression (Fig. 5A, B and 5C). We have also confirmed that BER inhibits the secretions of OPN and VEGF proteins (Fig. 6A and 6B) and MMP-9/MMP-2 mRNA (Fig. 7A and 7B) as well as activation of pro-matrix MMP-9/MMP-2 (Fig. 4C) in MDA-MB-231 cells. All these suppressions by BER are possibly involved in the reduction of the migration and invasion of MDA-MB-231 cells (Fig. 4A and 4B).

It should be noted that the breast cancer cell line MDA-MB-435S (parental cell line MDA-MB-435) used to be controversial a while ago but this cell line was employed in the present study. Ross et al., and G Ellison et al. suggested that MDA-MB-435 is a melanoma cell line [41,42]. However, from recent updating research, MDA-MB-435S is indeed a breast cancer cell line. The most convincing research is from the study by Sellappan S et al. [43]. They have demonstrated that the MDA-MB-435 is a breast cancer cell line since it expressed breast-specific milk components, including milk proteins and milk lipids, similar to that seen in MCF-7 breast cancer cells [43]. Also two very recent studies have firmly confirmed that MDA-MB-435 is a breast cancer cell line [44,45]. Many influential journals have also acknowledged that MDA-MB-435 is a breast cell line. For example, very recently, Kalaany and Sabatini have published their paper in *Nature *using MDA-MB-435 as a breast cancer cell line [46]. For these reasons mentioned above, we also applied MDA-MB-435S as a breast cancer cell line along with other breast cancer cell lines MDA-MB-231 and MCF-7 in the present study.

## Conclusion

By studying the activity of BER against human breast cancer cells and dissecting the molecular mechanisms of action of BER, we have demonstrated that BER significantly suppresses the in vitro and ex vivo growth of highly metastatic human breast cancer cells and enhances anticancer activity of anticancer agents celecoxib, trichostatin A and carmofur against the growth of MDA-MB-231 cells; BER also displays the strong activity of inducing apoptosis in both estrogen receptor-negative MDA-MB-231 cells and estrogen receptor-alpha-positive MCF-7 breast cancer cells. Down-regulation of Bcl-2 protein levels and up-regulation of pro-apoptotic Bax protein expression are possibly the one of important mechanisms of action of BER induced apoptosis in the cancer cell. BER also reduces the migration and invasion of MDA-MB-231 cells. In addition, we have confirmed that BER suppresses the Akt and NF-*κ*B signaling and their upstream target c-Met and downstream targets such as Bcl-2/Bax, OPN, VEGF, MMP-9 and MMP-2 in protein and/or mRNA levels in MDA-MB-231 cells, which are possibly associated with the suppression of growth, migration and invasion of MDA-MB-231 cells. Furthermore, BER shows synergistic effects with anticancer agents celecoxib, trichostatin A and carmofur on inhibiting the growth of MDA-MB-231 cells and reducing the ratio of Bcl-2/Bax and/or VEGF expressions in the cancer cells. All these findings suggest that BER may have the wide therapeutic and/or adjuvant application in the treatment of human breast cancer and other cancers.

## Methods

### Reagents

Berbamine (BER, molecular weight of 681.65, Fig 1A; purity greater than 99%) was purchased from Keji Pharmaceutical Co. (Liaoning, China) and dissolved in double distilled water (ddH_2_O) as a stock solution of berbamine. The series of working dilutions were made in DMEM cell culture medium. Matrigel and Boyden chambers were purchased from BD Inc. (Franklin Lakes, NJ) and Costar, Corning, Inc., (Corning, NY), respectively. Enhanced chemiluminescence Western blotting detection reagents were purchased from Amersham Pharmacia Biotech (Piscataway, NJ). Antibodies against Bcl-2, Bax, NF-*κ*B (p-65), Akt, p-Akt, c-Met, p-c-Met and β-Actin were purchased from Cell Signaling Technology, Inc. (Beverley, MA). Acrylamide and the protein assay kit were obtained from Bio-Rad (Hercules, CA). BER, trichostatin A (TSA or T), Ly294002 (LY), Bay 11-7082 (Bay), propidium iodide (PI), DMEM, penicillin, streptomycin, and 3- [4,5-Dimethylthiazol-2-yl]-2,5-diphenyltetrazolium bromide (MTT), trypsin/EDTA, fetal bovine serum, gelatin and all other chemicals employed in this study were purchased from Sigma Chemical Co. (St. Louis, MO). Celecoxib (S), carmofur (KA), navelbine (NA), rosiglitazone (Ro), and lovastatin (Lo) were obtained from Yuhuangding Hospital of Yantai, Yantai, Shandong Province, China.

### Animal experimentation and preparation of sera from BER-treated rats

SD rats (4 weeks old) were purchased from Luye Pharmaceutical Company, Yantai, Shandong, China. Animals were treated in accordance with guidelines established by the Animal Care and Use Committee at Yantai University. The animals were kept in animal facilities for at least one week before use, given water and a stock pellet diet (from the Luye Pharmaceutical Company) ad libitum, and kept in an air-conditioned room with an 8:00 a.m. to 8:00 p.m. light cycle. The preparation of sera from BER-treated rats was based on the methods of Zhang, et al. with slight modifications as described previously [47,48]. In brief, the rats were deprived of their diet at 6:00 p.m. but allowed free access to water until oral administration of BER which was conducted at 10:00 a.m. next day. BER was orally intubated to the rats at a dose of 10 mg/ml/100 g body weight. Blood samples were then collected at 0, 1, 2, and 3 h thereafter. The collected blood was left to clot for 2 h at room temperature and centrifuged twice at 3000× g at 4°C for 20 minutes. The sera were sterilized by filtration and then heated at 56°C for 30 minutes. The prepared sera were aliquoted, and stored at -80°C until ex vivo growth assay.

### Cell culture and in vitro and ex vivo growth assays

The highly-metastatic and estrogen receptor-negative human breast cancer cell lines MDA-MB-231 and MDA-MB-435S, and estrogen receptor-alpha-positive human breast cancer cell line MCF-7, and normal human mammary epithelial cell line MCF-10A were obtained from the American Type Culture Collection. MCF-7 cells were maintained in MEM supplemented with 0.1 mM nonessential amino acids, 1 mM sodium pyruvate, 1.5 g/L sodium bicarbonate, 10% fetal bovine serum, and antibiotics. The normal human mammary epithelial cell line MCF-10A was cultured in serum-free mammary epithelial growth medium (Clonetics, San Diego, CA) supplemented with 100 ng/mL cholera toxin (Calbiochem, La Jolla, CA). MDA-MB-231 and MDA-MB-435S were cultured in DMEM medium (Sigma, USA) containing 10% heat-inactivated fetal bovine serum, glutamine (2 mM), penicillin (100 U/ml) and streptomycin (100 μg/ml) at 37°C in a humidified incubator with 95% air/5% CO_2 _atmosphere. The *in vitro *and *ex vivo *assays were based on the methods of Zhang, et al. with slight modifications as described previously [47,48]. In brief, cells were cultured in the medium mentioned above supplemented with 10% FBS (in the case of *in vitro *assay) containing 0-80 μM BER alone or in combination with each anti-cancer agents (celecoxib, trichostatin A, carmofur, navelbine, rosiglitazone, lovastatin, Ly294002 and Bay 11-7082), or 10% rat sera (in the case of *ex vivo *assay) obtained at different time points after BER was orally intubated to rats. Cell growth was measured 24 h, 48 h (in the case of detection of the synergistic effects of BER and its anticancer agents), and 72 h after the treatments using 3-(4,5-dimethylthiazol-2-yl)-2,5-diphenyl-tetrazolium bromide (MTT) growth assay kit (Invitrogen) following the manufacturer's instruction. Each experiment was repeated three times.

### Flow cytometry for cell cycle analysis and apoptosis

The treatment of cells was based on the methods of Zhang, et al. as described previously [47]. MDA-MB-231, MDA-MB-435S, MCF-7 and MCF10A were treated for 48 h with BER at concentrations of 0, 20, 40, and 60 μM. The treated cells were detached in PBS/2 mM EDTA, centrifuged at 1,000 rpm for 5 min, and then gently resuspended in 250 μL of hypotonic fluorochrome solution (PBS, 50 μg propidium iodide, 0.1% sodium citrate, and 0.1% Triton X-100) with RNase A (100 unite/ml). The DNA content was analyzed by flow cytometry (Becton Dickinson FACS Vantage SE, San Jose, CA). Twenty-thousand events were analyzed per sample and the cell cycle distribution and apoptosis were determined based on DNA content and the sub-G_1 _cell population, respectively.

### In vitro migration and invasion assays

Tumor cell migration and invasion were measured by examining cell migration and invasion through fibronectin- and Matrigel-coated polycarbonate filters, respectively, using modified transwell chambers (Costar, Corning, Inc., Corning, NY). In brief, MDA-MB-231 cells (5 × 10^4^) were seeded onto the upper chamber in 200 μL of serum-free medium containing BER at the concentrations of 0, 1 μM, 10 μM, and 20 μM, respectively; the lower compartment was filled with 0.66 mL of DMEM media supplemented with 10% of FBS (as a chemo-attractant. After incubation for 6 h (in the case of migration assay) and 16 h (in the case of invasion assay) at 37°C, the cells that migrated or invaded to the lower surface of the filter were fixed and stained using propidium iodide. The cells on the upper side of the filter were removed using a cotton swab. The migrated or invaded cells on the underside of the filter were counted and recorded for images under a fluorescent microscope (Nikon, TE2000-U, Japan). Experiments were performed in triplicate.

### Gelatin zymography

The supernatants from the upper chamber of the transwell chamber in the aformentioned serum-free invasion assay were analyzed for pro-matrix metalloproteinase-9 (pro-MMP-9 or z-MMP-9) and pro-matrix metalloproteinase-2 (pro-MMP-2 or z-MMP-2) activation. The conditioned media were subjected to 10% SDS-PAGE containing 0.1% gelatin (under non-reducing conditions). Following electrophoresis, the gels were washed with 2.5% Triton X-100 to remove SDS and then incubated in a developing buffer [50 mM Tris-HCl buffer (pH 7.4), 10 mM CaCl_2_] overnight at 37°C. Gels were stained with 0.25% Coomassie Brilliant Blue R-250 and de-stained in the same solution without dye. Gelatinase activation was visualized as clear bands against the blue-stained gelatin background. Each experiment was repeated three times. The gelatin and all other chemicals were purchased from Sigma Chemical Co. (St. Louis, MO).

### Western blot analysis

This was performed according to our previous method [49]. In brief, MDA-MB-231 and MDA-MB-435S cells were treated with BER at the concentrations of 0 (0.1% DMSO vehicle as control), 40 μM, and 60 μM, and collected at 48 hours. For detection of effects of BER and its synergistic anticancer agents on Bcl-2 and Bax expressions in MDA-MB-231 cells, the cells were treated for 48 h with the indicated concentrations of BER (B, 20 μM), celecoxib (S, 20 μM), trichostatin A (T, 50 μg/L), Ly 294002 (LY, 25 μM), and Bay (5 μM) in the absence or presence of its synergistic anticancer agents S (20 μM), T (50 μg/L) and Ly (25 μM). For detection of p-Akt, the cells were treated for 30 minutes with BER at different concentrations. The treated cells were washed with ice-cold PBS and suspended in lysis buffer [20 mM Tris-Cl (pH 7.4), 100 mM NaCl, 1% NP40, 0.5% sodium deoxycholate, 5 mM MgCl_2_, 0.1 mM phenylmethylsulfonyl fluoride, 0.1 mM pepstatin A, 0.1 mM antipain, 0.1 mM chymostatin, 0.2 mM leupeptin, 10 μg/mL aprotinin, 0.5 mg/mL soybean trypsin inhibitor, and 1 mM benzamidine] on ice for 30 minutes. Lysates were cleared by centrifugation at 13000 rpm for 20 minutes. Equal amounts of cell extracts (60 μg) were resolved by SDS-PAGE, transferred to nitrocellulose membranes, and probed with primary antibodies to human Bcl-2, Bax, Nuclear factor (NF-*κ*B p-65), Akt, p-Akt, c-Met, p-c-Met and β-Actin and then horseradish-conjugated secondary antibodies, respectively. Anti-β-Actin antibody was used as a loading control. Detection was done using an enhanced chemiluminescence system (GE Healthcare Life Sciences).

### ELISAs for detection of human osteopontin and VEGF levels in human breast cancer cells

MDA-MB-231 and MDA-MB-435S cells were treated with BER at the concentrations of 0 (0.1% DMSO vehicle as control), 40 μM, and 60 μM for 16 h. For detection of effects of BER and its synergistic anticancer agents on the secretions of vascular endothelial growth factor (VEGF) in MDA-MB-231 cells, the cells were treated for 48 h with the indicated concentrations of BER (B, 10 μM, 20 μM and 40 μM), celecoxib (S, 10 μM, 20 μM, 40 μM, and 80 μM), trichostatin A (T, 25 μg/L, and 50 μg/L), carmofur (K, 40 mg/L), rosiglitazone (Ro1, 1 μM), lovastatin (Lo1, 1 μM), Ly294002 (LY, 25 μM), and Bay (5 μM) in the absence or presence of its synergistic anticancer agents K (40 mg/L) and T (25 μg/L and 50 μg/L). Then each supernatant of the cell culture was respectively collected and analyzed by ELISA using kits (osteopontin and VEGF) from R & D Systems, Minneapolis, MN. ELISAs were done according to the instructions of the manufacturer. Each experiment was repeated three times.

### Semi-quantitative reverse transcription-PCR

Total cellular RNA was extracted using TRIzol reagent (Invitrogen, USA) from MDA-MB-231 cells treated with BER at different concentrations (0/0.1% DMSO vehicle as control, 40 μM, and 60 μM) for 16 h according to the manufacturer's instructions, and quantified by spectrophotometry. RT reaction was done using total RNA as a template and a RT-for-PCR kit (Promega, Madison, WI). PCR amplification was carried out with the following primers:

MMP-2, 5'-GGATGATGCCTTTGCTCG-3' and 5'- CAGTGGACATGGCGGTCT-3'; MMP-9, 5'-TCCCTGGAGACCTGAGAACC-3' and 5'-GGCAAGTCTTCCGAGTAGTTT-3'; β-Actin, 5'-ATCATGTTTGAGACCTTCAACACC-3' and 5'-TAGCTCTTCTCCAGGGAGG-3'.

PCR conditions included an initial denaturation of 3 minutes at 94°C followed by 30 cycles of denaturation for 45 seconds at 94°C, annealing for 1 minute at 60°C, and extension for 1 minute at 72°C. Aliquots (10 μL) of the amplification products were separated by electrophoresis through a 1.5% agarose gel and visualized by ethidium bromide staining. The intensity of each band was quantified using Scion Image software (Scion, Frederick, MD). Results for each detected band intensity were normalized to β-Actin band intensity values. RNA only samples that gave completely negative results in PCR without reverse transcriptase were used to rule out the presence of genomic DNA contamination.

### Statistical analysis

The data were expressed as mean ± standard deviation (S.D.) and analyzed by the SPSS 13.0 software to evaluate the statistical difference. One-way or two-way ANOVA followed by the appropriate post hoc test (Bonferroni) was used to establish whether significant differences existed among groups. For confirming the synergistic effect between BER and each individual compound, comparison was made by two-way ANOVA followed by Bonferroni post hoc test. Values between different treatment groups at different times were compared. Mean concentrations and inhibition (%) are shown for each group; Asterisk *P *< 0.05, double asterisk *P *< 0.01, and triple asterisk *P *< 0.001. For all tests, *P *values less than 0.05 were considered statistically significant. All statistical tests were two-sided.

## List of abbreviation used

BER: berbamine; T: trichostatin A; LY: Ly294002; Bay: Bay 11-7082; S: celecoxib; K(A): carmofur; NA: navelbine; Ro: rosiglitazone; Lo: lovastatin; VEGF: vascular endothelial growth factor; pro-MMP-9: pro-matrix metalloproteinase-9; pro-MMP-2: pro-matrix metalloproteinase-2; OPN: osteopontin; COX-2: Cyclooxygenase-2; PI3K: phosphoinositide 3-kinase: NF-*κ*B: nuclear factor *κ*B; RT: reverse transcription; PCR: polymerase chain reaction.

## Competing interests

The authors declare that they have no competing interests.

## Authors' contributions

SW, QL, YZ, PY, KL, JL, HD, ZL and GZ performed the experiments, KL, FW, EW, KY and GZ analysed the data and prepared the manuscript, GZ designed the experiments and supervised the project. All authors read and approved the final manuscript.

*Shan Wang, Qian Liu, Ying Zhang, Ke Liu, and Pengfei Yu contributed equally to this work.
